This article has been retracted.

# Comparing the controlled attenuation parameter using FibroScan and attenuation imaging with ultrasound as a novel measurement for liver steatosis

**DOI:** 10.1371/journal.pone.0254892

**Published:** 2021-10-15

**Authors:** Po-Ke Hsu, Li-Sha Wu, Wei-Wen Su, Pei-Yuan Su, Yang-Yuan Chen, Yu-Chun Hsu, Hsu-Heng Yen, Chia-Lin Wu

**Affiliations:** 1 Department of Gastroenterology, Changhua Christian Hospital, Changhua County, Taiwan; 2 Institute of Medicine, Chung Shan Medical University, Taichung, Taiwan; 3 School of Medicine, Chung Shan Medical University, Taichung, Taiwan; 4 Department of Ultrasound, Changhua Christian Hospital, Changhua County, Taiwan; 5 Department of Nephrology, Changhua Christian Hospital, Changhua County, Taiwan; Kaohsiung Medical University Hospital, TAIWAN

## Abstract

**Background/Aims:**

In a recent study, attenuation imaging (ATI) with ultrasound was used as a new approach for detecting liver steatosis. However, although there are many studies on ATI and controlled attenuation parameter (CAP) that prove their practicability, there are few studies comparing these two methods. As such, this study compared CAP and ATI for the detection and evaluation of liver steatosis.

**Methods:**

A prospective analysis of 28 chronic liver disease patients who underwent liver biopsy, FibroScan® imaging, and ATI with ultrasound was conducted. The presence and degree of steatosis, as measured with the FibroScan® device and ATI, were compared with the pathological results obtained using liver biopsy.

**Results:**

The areas under the receiver operating characteristic curve (AUROC) of ATI and CAP for differentiating between normal and hepatic steatosis were 0.97 (95% confidence interval [CI] 0.83–1.00) and 0.96 (95% CI 0.81–0.99), respectively. ATI has a higher AUROC than CAP does in liver steatosis, at 0.99 (95% CI, 0.86–1.00) versus 0.91 (95% CI, 0.74–0.98) in grade ≥ 2 and 0.97 (95% CI, 0.82–1.00) versus 0.88 (95% CI, 0.70–0.97) in grade = 3, respectively.

**Conclusion:**

The ATI and CAP results showed good consistency and accuracy for the steatosis grading when compared with the liver biopsy results. Moreover, ATI is even better than CAP in patients with moderate or severe steatosis. Therefore, ATI represents a non-invasive and novel diagnostic tool with which to support the diagnosis of liver steatosis in clinical practice.

## Introduction

The diagnosis of liver steatosis is important to facilitate the treatment of chronic liver disease in clinical medicine [1]. Liver steatosis is generally considered to be a reversible and benign disease, yet researchers are increasingly attempting to reveal its role in the pathogenesis of various liver diseases [2, 3]. The development of fatty liver is related to steatohepatitis, and it can progress to liver fibrosis, cirrhosis, and even end-stage liver disease. In patients with chronic hepatitis C, liver steatosis accelerates the process of fibrosis [4–6], thus adversely affecting the sustained viral response rate of antiviral therapy [7, 8], and can predict the development of hepatocellular carcinoma due to liver steatosis [8, 9]. The evaluation of liver steatosis is also very important in the prognosis of liver transplantation donors because follicular steatosis of the donor liver is correlated with a risk of transplant failure after liver transplantation [10, 11].

According to the Clinical Practice Guidelines from the European Association for the Study of the Liver (EASL), the gold standard for the diagnosis and evaluation of fatty liver is liver biopsy [12], as the presence or absence of fatty liver and non-alcoholic fatty liver (NAFL) or non-alcoholic steatohepatitis (NASH) can only be distinguished by liver biopsy [13, 14]. However, this procedure is invasive and prone to triggering complications, such as pain, bleeding, and infection [15], and its results may be delayed due to the need to generate pathological reports. In addition, due to the high incidence of steatosis, its benign course, and the lack of clear association with liver enzyme changes, liver biopsy can only be deployed for some patients in need, such as in cases of non-alcoholic steatohepatitis, and because it is an invasive examination, it cannot be repeated, resulting in the inability to continuously and repeatedly monitor changes in patients with steatosis over a period of time.

Some studies have shown that using an ultrasound scanner such as FibroScan® (Echosens, Paris, France) together with the controlled attenuation parameter (CAP) can quantitatively and accurately assess the severity of liver steatosis in concordance with liver biopsy [16]. CAP estimates the total ultrasonic attenuation at the central frequency of the M probe or XL probe with FibroScan by using a go-and-return path [17]. However, FibroScan® is not an imaging device and cannot perform B-mode ultrasound assessments at the same time [18, 19].

In recent years, Canon Medical Systems has introduced an attenuation imaging (ATI) mode to the market as a novel ultrasound technique for diagnosing steatosis with the advantages of being easy to use and involving built-in ultrasonic machines [20]. ATI is a mode used to estimate the ultrasonic attenuation coefficient in tissues and can adjust the region of interest to measure liver attenuation and quantitatively evaluate liver steatosis through ultrasound imaging [21]. Based on two-dimensional images obtained in a daily ultrasound examination within a runtime of less than 2 minutes, ATI showed its convenience in routine screening of liver steatosis [22]. Compared with CAP, ATI’s advantage is the existence of an ultrasonic inspection mode; therefore, there is no need for additional equipment for examinations [23].

Another non-invasive tool is magnetic resonance imaging proton density fat fraction (MRI-PDFF), which can accurately quantify liver steatosis and provide a value of imaging diagnosis [24]. However, the cost of the instrument and the inconvenient operation are disadvantages [25, 26].

Given the current tools available for detecting liver steatosis, only few accurate, non-invasive, and easy-to-use detection methods other than CAP and ATI exist; therefore, this study aimed to compare the accuracy of CAP and ATI in assessing liver steatosis to support the identification of convenient and reliable methods for its clinical screening and treatment.

## Materials and methods

From January 1, 2019, to July 31, 2019, we prospectively included 48 patients with chronic hepatitis scheduled for liver biopsy at Changhua Christian Hospital who met the following study inclusion criteria: (1) age of 18 to 80 years; (2) body mass index of less than 35 but greater than 17 kg/m^2^; (3) signed the informed consent form. Meanwhile, the exclusion criteria were as follows: (1) malignancy, including hepatocellular carcinoma and cholangiocarcinoma; (2) chronic systematic disease, such as coronary artery disease, chronic kidney disease, and chronic respiratory disease; (3) alcohol consumption. The method of participant recruitment was the notification of liver biopsy from the hospital during this period. Once the patient provided signed consent, they were included in the study. Ultimately, 28 patients underwent liver biopsy, ATI, CAP assessment, and analysis. The demographic details of the participants show that they are all Asian and living in central Taiwan, mainly in the Changhua county. Moreover, all relevant data are within the paper. As stated, all participants signed an informed consent form for this study, which was reviewed and approved by the institutional review board of Changhua Christian Hospital (approval no. 210202).

### Liver biopsy

Under ultrasound guidance, a 16-gauge needle was used to obtain liver biopsy specimens. To be considered sufficient to score, the liver biopsy specimen had to measure at least 10 mm and have six portal tracts. The entire biopsy process was performed through percutaneous puncture over the right-side intercostal area of segments V-VI, and specimens were fixed with formalin, transferred to the pathology department of Changhua Christian Hospital within one hour [27], and stained with Masson’s trichrome. Meanwhile, reticulin staining was used to facilitate histological evaluation. All specimens were analyzed by two independent pathologists who were blinded to the clinical and laboratory characteristics of the patient under review. The steatosis grade was determined by the percentage of fat-containing cells in the liver sample that could be seen on a glass slide as follows: less than 5%, S0; 5% to 33%, S1; 34% to 66%, S2; and greater than 66%, S3.

### CAP measurement method

The CAP was measured by an experienced technician who did not know the patients’ clinical data, at the FibroScan^®^ facility, in dB/m. A 3.5-MHz standard probe (≥ 2.5 cm skin distance, XL probe; <2.5 cm skin distance, M probe) was used to measure the right liver lobe of the intercostal space while the patient lay on their back. The data reported by FibroScan^®^ had to meet the following conditions: (1) at least 10 effective shots, (2) a success rate of at least 60%, and (3) the interquartile range (IQR) was less than 30% of the median CAP.

### ATI measurement method

ATI was determined using data obtained from the TOSHIBA® i800 ultrasonic instrument (Toshiba, Tokyo, Japan) operated by a technician who did not know the results of the other reports. ATI allows for quantifying and color-coding changes in liver attenuation coefficients, which may be triggered by changes in the liver composition (e.g., increased fat content). The signal difference from point A to point B divided by the distance indicates the value of ATI, offering comprehensive quantitative data on liver steatosis (Fig 1). It also provides the slope of the signal attenuation (slope = attenuation coefficient). The value of ATI was defined as dB/cm/MHz × 100. The measurement was considered valid if the following criteria were met: (1) at least five effective values were collected, (2) a success rate of at least 60% was achieved, (3) an R^2^ value of 0.9 or greater at every single data point was recorded, and (4) the interquartile range was less than 30% of the median ATI.

**Fig 1:** Mechanism of attenuation imaging with ultrasound. The signal difference from point A to point B divided by the distance shows the value of attenuation imaging.

### Statistical analysis

First, we evaluated the normal distribution of the quantitative variables, in which the data are reported as mean and standard deviation values or median and interquartile range. The Kruskal–Wallis test, followed by the Dunn–Bonferroni post-test, was used to analyze the difference in the degree of ultrasound fatty liver between the four groups (S0, S1, S2, and S3). A two-tailed p-value of less than 0.05 was considered statistically significant.

The receiver operating characteristic curve (ROC) was used to evaluate the diagnostic performance of each non-invasive model. We calculated the area under the ROC curve (AUROC) and the 95% confidential interval (CI) of the AUROC. Then, using the De Long method, we compared the same data to judge the AUC value of different diagnostic criteria. We used Pearson’s correlation coefficient for ATI and CAP to confirm whether they are significantly related.

To evaluate the feasibility of the two measurements, we recalculated their diagnostic values (i.e., sensitivity, specificity, positive predictive value, and negative predictive value). These values were determined by original research. We used MedCalc statistical software version 19.4.0 (MedCalc Software Ltd., Ostend, Belgium; https://www.medcalc.org; 2020) for statistical analysis.

## Results

From January 2019 to July 2019, we included 48 patients with chronic liver disease scheduled for liver biopsy. Thereafter, four patients were excluded for malignancy, including hepatocellular carcinoma (n = 2) and cholangiocarcinoma (n = 2); furthermore, 11 were excluded for chronic systematic disease, such as coronary artery disease, chronic kidney disease, and chronic respiratory disease, and 5 were excluded for current alcohol consumption. Finally, 28 patients met the eligibility criteria for the following analysis (Fig 2).

**Fig 2:** Study flowchart.

The characteristics of the study participants are presented in Table 1. The patients had a mean age of 50.8 (± 14.0) years and eight (28.5%) were male. The risk factors for liver steatosis are baseline mean body mass index (BMI) value of 27.2 kg/m^2^, mean waist circumference of 89.4 cm, and diabetes mellitus (seven patients; 25%). The lipid profiles were as follows: mean triglyceride level: 149.0 mg/dL; cholesterol level: 188.2 mg/dL; high-density lipoprotein level: 50.4 mg/dL; low-density lipoprotein level: 125.2 mg/dL. Patient distribution according to steatosis grade was as follows: 6 (21.4%) patients with S0, 5 (17.8%) patients with S1, 9 (32.1%) patients with S2, and 8 (28.5%) patients with S3. The etiology distribution included 7 (25.0%) patients with hepatitis B virus infection, 9 (32.1%) patients with hepatitis C virus infection, 7 (25.0%) patients with nonalcoholic fatty liver disease, and 5 (17.8%) patients with autoimmune hepatitis; see Table 1.

**Table 1:** Clinical characteristics of the patients (n = 28).

Characteristic	Mean (±SD) or absolute count or median (interquartile range)
Age, years	50.8 ± 14.0
Male sex, n (%)	8 (28.5)
BMI, kg/m^2^	27.2 ± 3.8
Waist circumference (cm)	89.4 ± 12.8
Diabetes mellitus, n (%)	7 (25.0)
Triglyceride, mg/dL	149.0 ± 60.5
Cholesterol, mg/dL	188.2 ± 59.5
HDL, mg/dL	50.4 ± 20.2
LDL, mg/dL	125.2 ± 48.6
ALT, U/L	77.5 (34.3–125.8)
AST, U/L	56.5 (32.0–79.4)
Biopsy length, mm	16.5 ± 3.4
Liver stiffness, kPa	8.1 ± 2.3
Histology of steatosis grade*, n (%)	
S0	6 (21.4)
S1	5 (17.8)
S2	9 (32.1)
S3	8 (28.5)
Etiology of liver disease, n (%)	
HBV	7 (25.0)
HCV	9 (32.1)
NAFLD	7 (25.0)
AIH	5 (17.8)
ATI, dB/cm/MHz × 100	81.5 ± 14.1
CAP, dB/m	262.3 ± 51.1

AIH: autoimmune hepatitis; ALT: alanine transaminase; AST: aspartate transaminase; ATI: attenuation imaging; BMI: body mass index; CAP: controlled attenuation parameter; HBV: hepatitis B virus; HCV: hepatitis C virus; HDL: high-density lipoprotein; LDL: low-density lipoprotein; NAFLD: non-alcoholic fatty liver disease; SD: standard deviation

*Steatosis grade S0: <5%; S1: 5%–33%; S2: 34%–66%; S3: >66%

This study mainly compared the differences between the ATI and CAP assessment methods for liver steatosis of varying stages in patients with general chronic liver disease. The median (interquartile range) values for ATI and CAP according to liver steatosis grade were 67.5 (54.0–69.0) and 198.5 (193.0–206.0) for S0, 72 (72.0–78.5) and 261 (227.5–268.7) for S1, 82.0 (81.5–85.7) and 275 (255.7–283.5) for S2, and 98 (89.5–102) and 324.0 (290.0–338.0) for S3, respectively, with trends correlated to liver steatosis grading (p < 0.001, Jonckheere–Terpstra trend test); see Fig 3. ATI showed a significant difference in liver steatosis grading between S0 and S2, S0 and S3, and S1 and S3, with p < 0.05 in the post hoc analysis (Fig 3A), and CAP assessment showed the same result between S0 and S2 and S0 and S3, with p < 0.05 (Fig 3B). In addition, based on these data, ATI and the CAP were positively correlated (*r* = 0.8111; p < 0.05) (Fig 4).

**Fig 3:** The distribution of CAP and ATI values according to histologic steatosis grade. A: ATI was significantly different between S0 and S2, S0 and S3, and S1 and S3 (p < 0.05) with the Kruskal–Wallis test in the post hoc analysis. B: The CAP assessment results were significant between S0 and S2 and S0 and S3, with p < 0.05. The vertical axis is a logarithmic scale. The top and bottom of the boxes are the first and third quartiles, respectively. The length of each box represents the interquartile range, within which is located 50% of the values. The lines through the middle of the boxes represent median values. ATI: attenuation imaging; CAP: controlled attenuation parameter, *: p < 0.05.

**Fig 4:** The association between ATI and CAP. ATI and CAP were significantly correlated (r = 0.8111; p < 0.05).

We then analyzed the cut-off values of ATI and CAP to correctly predict steatosis. For this reason, we performed a comparative AUROC plot analysis, including all study participants (n = 28) with different steatosis grades. The AUROC of ATI according to liver steatosis grade was higher than that of CAP at 0.97 (0.83–1.00) to 0.96 (0.81–0.99) in S ≥ 1; 0.99 (0.86–1.00) to 0.91 (0.74–0.98) in S ≥ 2; and 0.97 (0.82–1.00) to 0.88 (0.70–0.97) in S3; see Fig 5. The sensitivity value that distinguished normal and liver steatosis (≥ S1) was 100% for ATI, which was higher than that of CAP at 95%. The positive predictive value (PPV) of CAP of 100% is higher than that of ATI of 95%, but the negative predictive value (NPV) of ATI of 100% is higher than that of CAP of 85%; see Table 2.

**Fig 5:** Comparing AUROC for ATI and CAP for detecting different grades of liver steatosis. A: Liver steatosis grade S1 or higher with AUROC values of 0.97 (95% CI: 0.83–1.00) for ATI (blue line) and 0.96 (95% CI: 0.81–0.99) for CAP (green line). B: Liver steatosis grade S2 or higher with AUROC values of 0.99 (95% CI: 0.86–1.00) for ATI and 0.91 (95% CI: 0.74–0.98) for CAP. C: Liver steatosis grade S3 with AUROC values of 0.97 (95% CI: 0.82–1.00) for ATI and 0.88 (95% CI: 0.70–0.97) for CAP. AUROC: area under the receiver operating characteristic curve; ATI: attenuation imaging; CAP: controlled attenuation parameter.

**Table 2:** CAP and ATI values for diagnosing liver steatosis.

Model	Steatosis stage	AUROC (95% CI)	Cutoff	Sen	Spe	PPV	NPV
CAP	S ≥ 1	0.96 (0.81–0.99)	220	0.95	1.00	1.00	0.85
	S ≥ 2	0.91 (0.74–0.98)	267	0.76	0.90	0.92	0.71
	S = 3	0.88 (0.70–0.97)	290	0.75	1.00	1.00	0.90
ATI	S ≥ 1	0.97 (0.83–1.00)	69	1.00	0.83	0.95	1.00
	S ≥ 2	0.99 (0.86–1.00)	78	1.00	0.90	0.94	1.00
	S = 3	0.97 (0.82–1.00)	82	1.00	0.85	0.72	1.00

ATI: attenuation imaging; AUROC: area under the receiver operating characteristic curve; CAP: controlled attenuation parameter; CI: confidence interval; NPV, negative predictive value; PPV, positive predictive value; Sen, sensitivity; Spe, specificity. Cut-off values were obtained from the original article.

## Discussion

In this study, the ATI and CAP values of mild and severe steatosis grades were found to increase significantly with increasing histologically diagnosed steatosis grade (p < 0.001, Jonckheere–Terpstra trend test). The AUROC values of ATI for diagnosing hepatic steatosis of grades S1 or higher, S2 or higher, and S3 were greater than those of CAP, suggesting that ATI is a more reliable method than CAP assessment for diagnosing liver steatosis.

Recent studies have suggested that CAP assessment via transient elastography (TE) can quantify the diagnosis of liver steatosis [17]. The CAP mode of TE is a non-image-based ultrasound technology able to measure the stiffness of tissues in real time and accurately [28]. Simultaneously, this technology can measure liver steatosis in CAP mode using M and XL probes; here, it revealed the AUROC for hepatic steatosis grades S1 or higher, S2 or higher, and S3 or higher to be 0.82 (95% CI 0.77–0.88), 0.83 (95% CI 0.77–0.88), and 0.89 (95% CI 0.84–0.93) for the M probe and 0.88 (95% CI 0.82–0.93), 0.92 (95% CI 0.89–0.96), and 0.93 (95% CI 0.89–0.97) for the XL probe, respectively [19]. Another study of patients with steatosis assessed by CAP showed an AUROC of 0.87 (95% CI 0.82–0.92) for S≥S1, 0.77 (95% CI 0.71–0.82) for S≥S2, and 0.70 (95% CI 0.64–0.75) for S = S3, and the Youden cut-off values of CAP for S≥S1, S≥S2, and S≥S3 were 302, 331, and 337 dB/m, respectively [29].

Another report showed that using the CAP mode of TE to detect liver steatosis in patients with hepatitis C presented AUROC values of 0.80 (95% CI 0.75–0.84) for S1 or higher, 0.86 (0.81–0.92) for S2 or higher, and 0.88 (0.73–1) for S3. CAP also exhibited a good ability to differentiate steatosis grades in hepatitis C patients (Obuchowski measure = 0.92) [30].

Compared with our study’s results, CAP yielded higher AUROC values in liver steatosis grades S1 or higher, S2 or higher, and S3. This result showed that CAP assessment could distinguish different grades of liver steatosis with a significant difference.

Recent studies have shown that, when comparing the measurement results for the proton density fat fraction based on magnetic resonance imaging with CAP assessment results based on TE, the former is more effective than CAP is in evaluating liver steatosis. A study showed that MRI-PDFF AUROCs for classifying steatosis grades 0 vs. 1–3, 0–1 vs. 2–3, and 0–2 vs. 3 were 0.98, 0.91, and 0.90, respectively [31]. Notably, ATI has a similar diagnostic mechanism in this study [32].

We acknowledge that there are several limitations to this study, including the small sample size, relatively obese patients (in patients with a BMI of 28 kg/m^2^ or more, CAP has no correlation with actual liver fat percentage) [33], patients being unblinded, possible selection bias in screening of patients, and other easily negligent and unobserved biases due to not using a randomized controlled clinical trial. The advantages of this study are as follows: (1) it is the first comparative study of ATI and CAP, (2) the prospective nature of the study with operators blinded makes the reports more credible, and (3) this study demonstrates that ATI is more reliable than CAP for diagnosing liver steatosis.

## Conclusions

ATI is a new method that is highly concordant with liver biopsy in detecting steatosis. ATI has a higher AUROC value in detecting different grades of liver steatosis than CAP, thus demonstrating ATI’s excellent and accurate diagnostic ability. In the future, ATI may be a promising technique for liver steatosis screening or diagnosis.

## Supporting information

S1 Data (XLSX)
